# Early Education Application Software Based on Artificial Intelligence VR Technology

This article has been retracted.

**DOI:** 10.1155/2022/4756390

**Published:** 2022-11-25

**Authors:** Zhengyue Zhao, Tongwei Xie, Huayi Wang, Yueyang Zheng

**Affiliations:** Kyungil University, Gyeongsan 38428, Republic of Korea

## Abstract

In order to solve the problems of restricted classroom and lack of repeated training in good curriculum, the design and development of a school life adaptation curriculum based on VR is proposed. This study identified six life adaptation themes for design and development (recognizing facial expressions, crossing the road, how to get lost, shopping, taking public transport, and job interview) and set the objectives, design principles, specific content, teaching evaluation, and other aspects of virtual reality life adaptation course. Combined with the characteristics of virtual reality, the implementation suggestions and matters needing attention are put forward. The results showed that, in the recognition of human facial expressions, 51 experts thought it was appropriate, 3 experts thought it needed to be modified, and no expert thought it was inappropriate. On the topic of crossing the road, 46 experts thought it was appropriate, eight thought it needed to be modified, and no expert thought it was inappropriate. On the theme of taking public transportation, 48 experts thought it was appropriate, 6 experts thought it needed to be modified, and no expert thought it was inappropriate. For the three major topics of how to get lost, shopping, and job interview, 2-3 experts put forward different opinions and think that the topic is not appropriate mainly because the grade arrangement is not appropriate. *Conclusion*. The VR-based curriculum for school life adaptation has been reviewed by experts and revised by researchers. It is scientific, interesting, and operable, solves the teaching problems of life adaptation teachers, and provides a safe, reliable, and effective practice channel for students.

## 1. Introduction

Virtual reality technology is one of the core contents of educational technology. The fundamental difference between virtual reality technology and other teaching methods is that virtual reality technology breaks the traditional teaching mode of one-way knowledge teaching. Students can give full play to their initiative and enthusiasm and enlighten 10 students on the fluency, flexibility, and delicacy of thinking. It provides abundant resources and convenient space for cultivating students' divergent thinking. It combines students' learning, practice, and self-test to form a vivid, lively, and active teaching method, which is beyond the reach of any traditional teaching method and method and has irreplaceable functions and effects [1]. Specifically speaking, the first is to have the special means of individualized teaching centered on students. The computer can give the learning content, instructions and questions, and other teaching information and can analyze and evaluate the learning effect according to the different solutions of students so that each student can be in a conducive to their own learning environment, with appropriate speed and multiple ideas and ways to answer questions. Second, the teaching form of virtual reality can make students choose the learning content suitable for their own difficulty and ease by observation and association according to their actual situation through a variety of sensory stimulation, so as to achieve the effect of teaching students in accordance with their aptitude. This way of learning provides students with a wider range of learning space and choice space and enhances their learning confidence. Third, virtual reality technology has interactive or man-machine dialogue characteristics. Virtual reality technology organically integrates teaching and practice so that students and computers are always in a series of alternating questioning and answering processes. In this kind of man-machine timely feedback dialogue process, students can be one or more, teaching mode can be diversified, teaching methods can be arbitrary, teaching speed can be multicontrolled, students can ask a question, a question to practice, and the computer provides a problem to solve, a changeable training function. In the process of training, students come into contact with many situations, find many problems, and propose many schemes, which broaden their thinking [2].

Virtual reality technology can also organically combine text, graphics, images, sounds, and animations and present them in front of students from all angles. This KIND of problem teaching method, heuristic teaching method, discussion teaching method, situational teaching method, suggestion teaching method, and discovery teaching method constantly stimulate the students' senses so that the students are in a state of excitement alternately through the brain regions. Thinking is fully active, arouses students' interest in learning, enriches students' imagination, and expands their thinking space. In the process of continuous increase and accumulation, creative inspiration and creative passion have been produced, and the train of thoughts has been broadened. Thinking produces flexibility, clarity, and fluency, thus cultivating students' divergent thinking and laying a good foundation for the cultivation of innovative thinking. In the discovery teaching practice, virtual reality can allow students to enter the environment where problems exist, construct virtual situations in a targeted and enlightening way, and guide students to explore. It uses a network structure form close to the characteristics of human cognition, and each node contains knowledge points of different media information. The logical link between each knowledge point constitutes the knowledge structure of the teaching content and provides a discovery learning thinking track [3]. Virtual reality teaching can not only provide good human-computer interaction but also allow students to make mistake so that students can understand the causes and consequences of mistakes and find the solution to the problem. Then, use advanced thinking skills such as analysis, comparison, induction, and reasoning to demonstrate the hypothesis, so as to approach or grasp the truth. Students develop discovery learning styles and strategies and develop high-level thinking skills. Virtual reality technology can construct the best classroom teaching environment and can provide and show a variety of realistic learning situations. Abstract learning is integrated with reality, so as to induce students' immediate thinking and stimulate students' associative thinking. Multimedia courseware has unique advantages in this regard, such as the use of computer simulation of university physics experiments in the electronic cloud. The rules of the movement of the electrons outside the nucleus are different from those of ordinary objects. They cannot be seen with the eyes and observed or measured with instruments, and there is no definite orbit for the movement of the electrons outside the nucleus. The operation speed is extremely fast, and the position of the electrons at a certain time cannot be seen, determined, and calculated. Only statistical methods can be used to describe the probability of the appearance of the exonuclear electron in a certain region of space outside the nucleus. Therefore, the content is very abstract and difficult for teachers and students to teach as shown in Figure 1.

## 2. Literature Review

Rohani et al. proposed that, in the development and application of virtual reality technology, more attention should be paid to the application in the field of education, which is the cradle of creating talents. If virtual reality technology can be applied to build corresponding scenarios, it will also greatly promote the development of VR technology in the future [4]. Segura et al. proposed to build a physical laboratory by applying virtual reality technology to make up for the limited operating environment in educational classrooms [5]. This research proposal has also received a great response in Malaysia. Through the construction of interactive virtual reality scenes, students' understanding of speed in physics teaching is more specific. Although the UK's research on the application and development of virtual reality technology started later than that of the United States, it paid more attention to the sensory construction of interactive scenes in its research. On the basis of simple visual experience, it also introduced vision, touch, and even smell. When people experience virtual reality interactive scenes, they have a sense of environmental substitution. Puggioni et al. proposed that the development of virtual reality technology should be conducted from the perspective of the combination of software and hardware. What software development creates is only a visual scene, and the combination of hardware and software can mobilize different sensory stimuli to form a more specific scene [6]. This research proposal has a great inspiration for the research of virtual reality technology in China. At the early stage of its development, China's virtual reality technology fully drew on the existing research results of foreign countries. Rafique and Cheung built the human science museum through the application of virtual reality technology, so as to carry out more specific reform of medical teaching [7]. The application of virtual reality technology in different fields will also determine the development focus. The application research of virtual reality technology in China has now entered the stage of visual sensory optimization, and future development will focus on the mobilization and development of multiple sensory worlds. Kami ń Ska's et al. experimental research on the direct learning ability and strategies of 4–6-year-old children shows that children have sprouted the direct learning ability under language conditions, but the age development effect is not obvious, and many strategies coexist in children's direct reasoning [8]. For example, children's knowledge of logarithms cannot be obtained through direct perception like their knowledge of size and color, but through an abstract process. Children's acquisition of mathematical knowledge is not through direct perception, but through the coordination of a series of actions. Konrad et al. tested the spatial cognition and learning ability of 4–7-year-old children and concluded that the rapid improvement period of cognitive performance of children's learning ability occurred in the 5 months (initial enrollment) from the age of 7 to 7 years [9].

Gong et al. carried out an experiment on the reasoning ability of children aged 5-6 years. The experiment proved that children at this age have the ability to initially understand the transitivity in quantity, which is also a good period to understand the transitivity. Children's cognitive structure has transitivity, and they also have learning ability [10]. Adwernat et al. combined with his own research and published a paper “the ultimate display” on virtual reality technology, proposing that the computer screen the authors use can actually act as a window to view the virtual reality world, and it is this idea that has inspired people's research boom on virtual reality technology [11]. After several years of efforts, Serrano Vergel et al. finally developed the ultimate display and named it the sword of Damocles. The display contains two CRT displays, through which more images can be displayed. At the same time, the device also includes mechanical links and ultrasonic detectors so that users can complete control through handheld terminals, thus realizing interaction with the virtual reality world [12].

Combining with the practical problems encountered by front-line teachers in special education in life adaptation teaching, a virtual reality life adaptation curriculum intervention system suitable for students in a school in China is independently developed and designed in this essay. Through long-term teaching and training, it verifies to what extent special children in a school can benefit from virtual reality intervention. The developed virtual reality intervention system will be applied to the learning of students in a school through the long-term teaching of life adaptation teachers, and the best intervention mode of VR will be explored in combination with the obstacle level of students. This will help cultivate the independent living ability of students in a school and help them better adapt to society.

## 3. Research Methods

The research methods are explained in the following sections.

### 3.1. Virtual Reality Life Adaptation Course Goal Setting

According to the curriculum standard for life adaptation in compulsory education of a school (2016 Edition), the overall goal of a life adaptation curriculum is to help students understand basic life knowledge, master necessary adaptive skills, develop good behavior habits, and form basic life adaptation ability and good morality [13–16]. Under the principle of abiding by the overall goal, in combination with the suggestions and guidance of life adaptation teachers, specific objectives of VR-based life adaptation theme teaching are proposed, as shown in Table 1.

### 3.2. VR Life Adaptation Course Theme Classification Design

A total of six life adaptation teaching topics were selected for the following reasons. First, the interview with life adaptation teachers found that these six life adaptation teaching topics could not provide students with practice opportunities in the actual teaching process, resulting in poor classroom effect, and belong to the top ten life adaptation teaching problems in the teaching of a school. Second, these six life adaptation teaching topics cover the low, middle, and high stages of a school, which are closely related to the daily life of students, and are of great significance to the development of students at each stage. Third, overseas VR practice teaching has given us sufficient confidence [13]. The learning of life skills is a systematic learning, and each subject can neither be learned overnight nor can be learned in one grade [17–19]. Therefore, in actual teaching, grade adjustment should be made according to individual development level, or teaching progress should be adjusted according to students' acceptance.

#### 3.2.1. Recognizing Facial Expressions (Grade 2 and Grade 3)

Recognition of human facial expressions is the learning content of the lower grades in a school, and recognition of human emotions is the basis and premise for students to engage in social communication with others [20, 21]. However, most of the students in a school have difficulties in learning to recognize human facial expressions, especially autistic students, who experience emotions such as happiness, grief, and fear in VR. Students gradually learn to express their emotions appropriately on appropriate occasions [14]. After students recognize the expressions of anger and fear in the first part, they enter into the practice session. After participating in the last six parts, students choose the corresponding expressions (the face is covered by the Mosaic effect and the correct choice will be shown).

#### 3.2.2. Crossing the Road (Grade 3)

Crossing the road safely is the learning content of students in low, middle, and grade levels in a school. When training students in VR to cross the road, students' obstacle degree should be taken into account, and teaching should be conducted according to the obstacle degree and actual needs of students. The arrangement of grades can be adjusted appropriately [22–25].

(1) Stage 1 (no traffic lights and no zebra crossings): at the intersection without traffic lights and zebra crossings (there are only two buildings in the southeast and southwest directions of the intersection, which can be supermarkets, hospitals, shopping malls, exhibition halls, libraries, bookstores, restaurants, convenience stores, etc.), there is only a small car coming to the left front of the subject, and the speed is very slow (the car can be seen within the subject's vision range). It was a long distance away from the subjects and the vehicle speed was very low. It was observed whether the subjects waited for the vehicles to pass before crossing the road or straight across the road, recorded the reaction time of the subjects when crossing the road, and whether the subjects flinched when crossing the road [15], as shown in Table 2.

(2) Stage 2 (no traffic light and zebra crossing intersection): at the intersection with no traffic light and zebra crossing (there are 6 buildings in all directions of the intersection, which are relatively few, such as supermarkets, hospitals, shopping malls, exhibition halls, libraries, bookstores, restaurants, and convenience stores,), and on each street, there are one or two cars coming and going, most of which are very slow, but there is a slightly faster one, and there are a few pedestrians (2-3 people). We observe whether the subjects wait for the vehicles to pass before crossing the road safely on the zebra crossing [26–29]. The reaction times of the participants were recorded, as well as whether the participants flinched when crossing the road, as shown in Table 3.

(3) Stage 3 (intersection with traffic light and zebra crossing): at the intersection with traffic lights and zebra crossing (there are all kinds of tall buildings in each direction of the intersection, which can be supermarkets, hospitals, shopping malls, exhibition halls, libraries, bookstores, restaurants, and convenience stores,), there are also many cars, buses, electric cars, and tricycles, (in different colors, shapes, and sizes) on the four-way streets. The speed is urgent and slow, and there are many pedestrians [30–32]. Observe whether the subjects wait for the green light to turn on and then pass the zebra crossing safely after the traffic passes [16]. The reaction times of the participants were recorded; whether the participants flinched when crossing the road was also recorded, as shown in Table 4.

(4) Phase four (two consecutive intersections): two consecutive intersections were 50 m apart. The first intersection was traffic light without zebra crossing (there are all kinds of tall buildings in all directions of the intersection, which are all over the dense, and can be supermarkets, hospitals, shopping malls, exhibition halls, libraries, bookstores, restaurants, convenience stores, etc.). There are two or three cars, buses, electric cars, etc. (of different colors, shapes, and sizes) in a four-way street, and the speed is relatively slow [33, 34]. There were 5-6 pedestrians, and the participants were observed whether they waited for the green light to turn on and the traffic to pass before crossing the road safely. The reaction times of the participants were recorded; whether the participants flinched when crossing the road was also recorded.

When the subject passes the first intersection safely, he is guided to the next intersection safely through the voice prompt. At the second intersection, there are traffic lights and zebra crossings (there are all kinds of tall buildings in all directions of the intersection, which are very dense and can be supermarkets, hospitals, shopping malls, exhibition halls, libraries, bookstores, restaurants, convenience stores, etc.). There are many cars, buses, electric cars, etc. (in different colors, shapes, and sizes) on the four-way street. The speed is urgent and slow, and there are many pedestrians. We observe whether the subjects wait for the vehicles to pass and whether they wait for the green light to turn on before safely crossing the zebra crossing road [17]. The reaction times of the participants were recorded; whether the participants flinched when crossing the road was also recorded, as shown in Table 5.

#### 3.2.3. What to Do If You Get Lost (Mayday 4th Grade)?

According to Curriculum Standards (2016 edition), life adaptation courses in middle grade are based on families, schools, and communities, focusing on cultivating students' ability to do simple housework, forming self-protection awareness, and guiding students to develop independently. The students in the middle grade of compulsory education in a school have the most basic self-care ability, and the demand for social communication is gradually increasing, and the opportunities for outdoor activities are increasing [35–38]. Through interviews with life-adapted teachers and personal participation in classroom practice, it is found that, in the teaching process of this stage, there are the biggest difficulties in the actual teaching process of how to do when lost, shopping in supermarkets, and taking buses [18]. The teaching problems in the middle grade should also be taught in VR according to the degree of obstacles and actual needs of students, and the arrangement of grades can be adjusted appropriately.

#### 3.2.4. Shopping (Grade 4)

Shopping in the supermarket is closely related to students' life. Students in a certain school lack the opportunity to practice and exercise and do not know the process of shopping and matters needing attention.

Before going shopping, users first list what they need to buy and enter the virtual reality with a purpose.

When they come to the supermarket to prepare for shopping, the VR situation initially appears at the entrance of the supermarket. Users participate in the VR situation and enter the supermarket by following the guidance of the road signs. They go to the shelves and choose one by one according to the shopping list they have made.

The user follows the guide to the target shelf, finds the desired item, and continues to find the remaining items (or find them by themselves) in accordance with this method.

After shopping, after all the desired items have been selected, the user goes to the supermarket exit to line up the checkout. There are four checkout Windows, and at three, there are many people in line. The number of people in the queue at 1 window is small, and the user needs to queue up to check out (if he does not queue up, he will get automatic feedback from the system, such as you can't jump the queue! The system's voice instructs users to queue in order. When the user pays, the cashier asks the user:

  Cashier: hello, your total charge is 50 yuan. Would you like to pay in cash or online?
  User: pay online (show the payment code to the cashier). Or if the user's ability permits, pay in cash and get the change.
  Cashier: thank you. You have paid. Please bring everything you bought.
  User: thank you.
  End of shopping learning in VR context.

#### 3.2.5. Taking the Bus (Grade 5)

Taking the bus is what middle-grade students in a school learn. The main design ideas are as follows: for medium-sized buses, the appearance and size of buses are the same in the four stages of taking buses, and each stage is only distinguished by color. There are 30 seats in the bus, and the seats in the car, the color of the car, and the passengers should be distinguished. The bus driver's seat, steering wheel, windshield, and other stages are different.

(1) Stage 1 (a quiet, empty bus with no one waiting in line): the user waits for the bus at the bus station alone. When the bus arrives, the door opens, and the bus is empty. After swiping the card, the user enters the bus, and all the seats in the front, middle, and back rows are empty.

(2) Stage 2 (a bus with queues, a bit of noise, and a few passengers): when the user arrives at the bus station, there are 5 people waiting in line for the bus. According to the voice prompt in the VR situation and the association with the classroom teaching, the user voluntarily waits in line for the bus at the bus station (if they are not in line, they will get automatic feedback from the system, such as you can't cut in line! Then instruct them to react accordingly in order). When the car arrives, the door opens. With five passengers on board, users line up to swipe their cards to get on the bus. There were 11 passengers in the carriage, which was relatively small. There were still empty seats in the front, middle, and back rows of the bus, and some seats were filled with bags and other items. The user chooses the seat according to his own preference (if the user does not take the initiative to find a seat to sit down, a voice prompt will appear: on a crowded bus, the user can ask if he can sit in the seat with the bag). If the user chooses the seat without the bag, he can sit down directly. If you choose a seat next to a passenger with a bag, you need to get permission from the passenger first.

(3) Stage 3 (buses with queues, noisy compartments, and lots of passengers): when the user arrives at the bus stop, there are already 10 people waiting in line for the bus. According to the voice prompts in the VR situation and the association of classroom teaching, users voluntarily queue up at the bus station to wait for the bus (if they are not in the queue, they will get automatic feedback from the system, such as you cannot cut in line! Then instruct them to react accordingly in order). When the car arrives, the door opens. With 10 passengers on board, users lined up to swipe their cards to get on the bus. There were 21 passengers in the carriage, which was relatively large. There are only empty seats in the middle row and the back row of the bus, but these seats are basically filled with bags and other items. Users can choose the seat according to their own preferences (if the user does not take the initiative to find a seat, the voice prompts: let him ask if he can sit in the seat with the bag on the crowded bus). If you choose a seat next to a passenger with a bag, you need to get the consent of the passenger first, as shown in Table 6.

#### 3.2.6. Interview (Secondary School)

According to the Curriculum Standards (2016 edition), the curriculum of life adaptation in senior grades penetrates the understanding of society, family, and the world and focuses on developing the ability of self-protection and social adaptation, cultivating a positive and optimistic attitude towards life, so that students can live a safe and healthy life. Through interviews with teachers adapting to life, it is found that the core teaching theme of the senior stage is centered on work. The main contents include understanding common professionals (doctors and police), and students may be engaged in future career (packers, cleaners, catering, and waiters), cultivating students' consciousness of labor and labor quality (to insist, be patient, to be punctual, obey the arrangement, working with people, understanding the labor remuneration, and dry), and leading the students to participate in the internship practice (asylum to the factory to study Packers, to do cleaning work in the hotel, to the supermarket as a supermarket tally clerk, to the restaurant as a waiter, learn nail art, and learn beading). According to the life adaptation teachers, some graduates with better abilities from a certain school have been assessed by the employing unit after graduation, and indeed some students are engaged in these jobs. The graduates of a school are mostly engaged in simple repetitive work, which does not require deep knowledge, so they basically do not need to go through the tedious interview process. However, to establish a connection between workers and employers and finally determine the employment of workers, they still need to communicate with employers to leave a good impression on employers. Informal interviews between workers and employers are particularly necessary. In order to help life adaptation teachers' professional teaching in senior grades and to make the job interview of graduates of a school more smooth, VR job search training is designed to exercise the interview skills of senior students. Considering that some schools do not offer vocational education courses, the content of this stage can be arranged in the senior stage, and for schools with vocational education courses, it can also be arranged in the vocational education stage.

Before entering the VR job training system, users fill in relevant personal information through an online application, such as education experience, internship experience, and special skills, and then enter positive communication with the interviewer to train the whole interview process.

In VR, the user answers different questions raised by the interviewer, which are mainly aimed at correcting errors. If the user has inappropriate replies or fails to answer any questions, he/she can master some interview skills through repeated practice and gradually improve his/her interview level.

In the VR job training system, the interviewer finished asking questions and entered the fourth link one by one.

### 3.3. Learning Evaluation of VR Life Adaptation Course

The purpose of VR-based life adaptation course is to cultivate students' basic life skills and improve their ability to live independently. Due to the intelligence defects of students in a school, their acquisition of knowledge or skills often goes through a long process, requiring many exercises and practices. Therefore, life adaptation teachers need to establish “one person, one case” in the process of practical teaching. Before practicing in VR, students should be tested first to ensure that students have no adverse reactions in VR and are initially familiar with the VR environment. In practice, students' learning process in VR should be recorded and evaluated (formative evaluation). Refer to Tables 7–12 for evaluation.

### 3.4. Network Latency

In order to overcome the influence of the dynamic change of network on data transmission, network QoS monitoring technology is introduced, and real-time monitoring is used to lay a good foundation for intelligent transmission control. We add a timestamp to the protocol layer to monitor the network delay. We add two fields to each packet to record the last received timestamp (LRT) and the current sent timestamp (CST). After receiving the packet, the receiver calculates the local packet sending delay based on the LRT and SCT of the packet. At the same time, the processing delay of the packet in the network can be obtained by subtracting the processing delay of the peer end based on the saved last packet sending timestamp (LST) and the received packet time at the receiving end.

When end B sends A reply to End A, (1) and (2)areas follows:

(1) $$\begin{array}{c} LRT=TB+∆t1\text{,} \end{array}$$

(2) $$\begin{array}{c} CST=TB+∆t1+∆t2\text{.} \end{array}$$

When end A receives a packet from end B, its local formula is as follows:

(3) $$\begin{array}{c} LRT=TA+∆t1\text{.} \end{array}$$

Moreover, its current time is shown as follows:

(4) $$\begin{array}{c} CT=TA+∆t1+∆t2+∆t3\text{.} \end{array}$$

In this case, the bidirectional delay of packet sending can be calculated as follows:

(5) $$\begin{array}{c} CT-LST-\left(CST-LRT\right)\text{.} \end{array}$$

## 4. Results' Analysis

### 4.1. Topic Selection

The data obtained from the survey were input into SPSS and analyzed. In the choice of the theme of the VR life adaptation course, 54 experts agreed that the theme of the VR life adaptation course was suitable for the learning of students in a certain school. When it comes to recognizing facial expressions, 51 experts said they were appropriate, three said they needed to be modified, and none said they were inappropriate. On the theme of road crossing, 46 experts think it is appropriate, 8 experts think it needs to be modified, and no expert thinks it is inappropriate [19]. On the theme of taking public transportation, 48 experts thought it was appropriate, 6 experts thought it needed to be modified, and no expert thought it was inappropriate. For the three major topics of how to do lost, shopping, and job interview, 2-3 experts put forward different opinions and think that the topic is not appropriate mainly because of the grade arrangement is not appropriate. Experts suggest that the topic of what to do when lost should be taught at every grade level. Shopping is a topic that should be studied in the fifth or sixth grade. Job interviews should be studied in vocational education. See Figure 2 for details as follows:

### 4.2. Target Setting

The data obtained from the survey were input into SPSS and analyzed. On the goal setting of the VR life adaptation course, the opinions of experts are also relatively consistent, and most of them think that the goal setting of the VR life adaptation course is suitable for students in a certain school. However, some experts put forward suggestions for modification, believing that the setting of some curriculum objectives is not specific enough, and it is difficult to implement in the actual implementation [20]. As for the modification opinions put forward by experts, the reasonable part is absorbed, and the goal setting of some life adaptation courses is modified to complete this part. The expert opinions are detailed in Figure 3 as follows.

### 4.3. Evaluation System

On the evaluation system of the VR life adaptation course, the opinions of experts are also relatively consistent, and they believe that the evaluation system of the VR life adaptation course is suitable for the learning evaluation of students in a certain school. In the five major topics of recognizing facial expressions, crossing the road, how to get lost, shopping, and taking public transport, experts did not put forward inappropriate opinions. Only on the topic of a job interview, one expert puts forward inappropriate modification opinions. The evaluation system of the virtual reality life adaptation course was modified according to the modification opinions put forward by experts. For details, see Figure 4.

## 5. Conclusion

The curriculum design of a school life adaptation based on VR has been reviewed by special education experts, curriculum theory experts, and virtual reality technology experts and revised by researchers. It is scientific, interesting, and operable, solves the teaching problems of life adaptation teachers, and provides a safe, reliable, and effective practice channel for students.

For future research, it can be further improved when time permits. First of all, the selection of interview objects should be different, that is, taking into account the life adaptation teachers in different regions, levels, and stages, and ensuring the comprehensive content of the interview. Secondly, the authors should consider the needs of teachers as comprehensively as possible when the authors design and develop the problems of life adaptation teaching in various stages of cultivating wisdom schools. The teaching topics which are difficult to adapt to life mentioned by teachers are analyzed scientifically to see whether these topics are suitable for the development of auxiliary teaching in the form of VR. Further research will be carried out on topics that are suitable for the development of ADT in the form of VR. Finally, at present, only the teaching topic of crossing the road has been developed. It is necessary to accelerate the development of other VR-based life adaptation courses and put them into use to help teachers adapt to living.

## Figures and Tables

**Figure 1:** Artificial intelligence VR technology.

**Figure 2:** Experts' evaluation of the appropriateness of topic selection.

**Figure 3:** Experts' evaluation of the appropriateness of goal setting.

**Figure 4:** Experts' evaluation of the appropriateness of the evaluation system.

**Table 1:** Objectives of virtual reality life adaptation course.

VR life adaptation course topic classification	Specific goals
Recognize facial expressions	Teaching objectives: to perceive people's emotions such as happiness, sorrow, and fear in specific situations and to know the existence of emotions, learn to distinguish people's emotions such as anger, sorrow, and fear, grasp the meaning of several basic emotions, and learn how to use basic emotions in specific situations
	Ability objectives: obey the teacher's instructions, actively participate in class activities, and learn people's emotions through VR; according to the specific situation in VR, students can learn the expression ways of certain emotions, and the teachers can guide students to gradually learn the transition from virtual to reality

Cross the road	Teaching objectives: to understand traffic lights, zebra crossings, pedestrian bridges, and road signs, understand the traffic rules: stop at the red light, go at the green light, and wait when the yellow light is on; if the left side cannot be crossed, then go right, look around, and cross slowly; zebra crossing is the safest
	Ability objective: obey the teacher's instructions, master the precautions for crossing the road, and learn how to cross the road safely in different situations through VR, in VR, I can obey the traffic rules: stop at the red light, go at the green light, and wait when the yellow light is on; if the left side cannot be crossed, then go right, look around, pass slowly, and the zebra crossing is the safest, so I can cross the road safely; after practicing several times in VR, cooperate with parents; under the condition of ensuring the safety of students, students gradually learn to cross the road at actual junctions

What if I get lost	Teaching goals: know your name and school and know the exact location of your home Ability objective: in VR situation, when lost, I cannot panic and actively seek help, can recite the location of their home, parents, and other people's contact information or take the initiative to show their own information card, be able to ask for help from police, security personnel, etc.

Shopping	Teaching objectives: understand the supermarket and know the function of the supermarket, master the basic process of shopping: bring your mobile phone or prepare the money, choose whether to deposit or withdraw the bag at the entrance, enter the supermarket from the entrance, select the items you need and like, go to the cashier to line up, arrange the bought items into the bag, and retrieve the things you deposit and leave
	Ability objective: to obey the teacher's instructions and master the shopping rules in VR; after practicing in VR many times and cooperating with parents, students gradually learn how to shop in an orderly and civilized way in a real supermarket

Taking the bus	Teaching objectives: to know the bus; master the process of taking the bus: queue up, swipe the card, find a seat, wait for the arrival hint, and get off the bus
	Ability objective: obey the teacher's instructions, master the precautions for taking public transport in VR, and learn how to take public transport in different situations through VR; after practicing in VR many times and cooperating with parents, the students gradually learned to cope with different bus environments by themselves when they went out to take their children by bus

Finding a Job interview	Teaching objectives: to understand some common occupations and form a sense of rewarding labor, in appearance, the appearance is neat and well-dressed, show a friendly interview attitude, smile, communicate in an honest manner, and show respect to the interviewer
	Ability goals: learn how to introduce yourself to the interviewer, learn how to present your strengths to the interviewer, and actively answer the interviewer's questions without flinching; after practicing in VR many times, accompanied by parents and teachers, I can actively cope with the real interview situation and leave a good impression on the interviewer

**Table 2:** Intersection without a traffic light and zebra crossing.

The main project	Project indicators
The crossroads	There are only Z buildings, all kinds of landmarks, trees, guardrails on both sides of the road, streets, and sidewalks in the southeast and southwest directions of the intersection
Number of vehicles	Each driving direction has 1 vehicle and a total of 4 quantities
The speed of the car	10 km/h
Number of passengers	One person on the opposite side and only one person on the subject's side
Distractors	The car
Sound	Car horns
Other interference	None
The weather conditions	A sunny day with moderate temperature

**Table 3:** Crossings without traffic lights and zebra crossings.

The main project	Project indicators
The crossroads	There are all kinds of tall buildings, all kinds of road signs, trees, guardrails on both sides of the road, streets, sidewalks, and S buildings
Number of vehicles	Each driving direction has 1 or two vehicles and a total of 6 vehicles
The speed of the car	15 km/h
Number of passengers	On both sides of the zebra crossing, about 2-3 people on each side
Distractors	Vehicles (cars or buses, or electric cars, or tricycles), pedestrians, and road signs
Sound	The sound of car sirens and the noise of people going and going
Other interference	None
The weather conditions	A sunny day with moderate temperature

**Table 4:** Intersection with a traffic light and zebra crossing.

The main project	Project indicators
The crossroads	There are all kinds of tall buildings, all kinds of road signs, trees, guardrails on both sides of the road, streets, sidewalks, and a total of 10 buildings
Number of vehicles	Each driving direction has 1 or two vehicles and a total of 12 vehicles
The speed of the car	20 km/h
Number of passengers	On both sides of the zebra crossing and about 3-4 people on each side
Distractors	Vehicles (cars or buses, or electric cars, or tricycles), pedestrians, and road signs
Sound	The sound of car sirens and the noise of people going and going
Other interference	None
The weather conditions	A sunny day with moderate temperature

**Table 5:** Two consecutive intersections.

	The main project	Project indicators
At the first crossing	The crossroads	There are all kinds of tall buildings, all kinds of road signs, trees, guardrails on both sides of the road, streets, sidewalks, buildings all over very dense, and 8 buildings
	Number of vehicles	Each driving direction has two or three vehicles and a total of 10 vehicles
	The speed of the car	20 km/h
	Number of passengers	On both sides of the crossing and about 5 people are on each side
	Distractors	Vehicles (cars or buses, or electric cars, or tricycles), pedestrians, and road signs
	Sound	The sound of car sirens and the noise of people going and going
	Other interference	Two crossings

At the second crossing	The crossroads	There are all kinds of tall buildings, all kinds of road signs, trees, guardrails on both sides of the road, streets, sidewalks, very dense buildings, and 12 buildings
	Number of vehicles	Each driving direction has four vehicles and a total of 16 vehicles
	The speed of the car	25 km/h
	Number of passengers	On both sides of the crossing and about 5-6 people are on each side
	Distractors	Vehicles (cars or buses, or electric cars, or tricycles), pedestrians, and road signs
	Sound	The sound of car sirens and the noise of people going and going

**Table 6:** Project index reference at each stage of the bus ride.

	The number of line	The car environment	The number of people in the car	Are there any seats available?	Do you need to ask?
Stage 1	1 person	Quiet	0	Yes, it is completely empty	No
Stage 2	6 people	A bit noisy	5 people	Yes, more seats	According to the choice of subjects
Stage 3	I1 people	More noisy	10 people	Yes, there are fewer vacancies	Yes
Stage 4	16 people	Very noisy	25 people	There is no vacancy	According to the situation on the bus

**Table 7:** Recognizing others' facial expressions: student learning evaluation record.

	Evaluation of project	Score		
		2 points	1 point	0 point
		The student just chooses the right answer	There was hesitation, thought for a long time, but the student eventually came up with the right answer	After thinking for a long time, the student cannot give the right answer or give the wrong answer directly
The first practice	To experience joy			
	Feel sad			
	Feel the anger			
	Experience surprise			
	…			

The second practice	To experience joy			
	Feel sad			
	Feel the anger			
	Experience surprise			
…	…			

**Table 8:** Students' learning evaluation form crossing the road.

Evaluation of project	Score			
	3 points	2 points	1 point	0 point
Whether to observe the traffic lights before crossing the street	The student was able to observe traffic lights independently and within 5′ before crossing the road	The student was able to observe the traffic lights independently before crossing the road but take more than 5′	He has no awareness of observing traffic lights independently before crossing the road, but he can observe traffic lights after being reminded	After the warning, he still crossed the road without observing the traffic lights

Reaction time to start crossing the street when the light turns green	The time is within 0–5	The time is within 5.1–10'	It's within 10–15′	Time over 15′

Whether to walk on a zebra crossing	The student was able to cross the road independently and walk on the zebra crossing the whole time	The student was able to cross the road independently, but not on the zebra crossing the whole time, such as initially walking on the zebra crossing and then deviating from the zebra crossing or initially deviating from the zebra crossing and then walking on the zebra crossing	The student was not able to cross the road independently, but after reminding, can walk on the zebra crossing	The student still walked outside the zebra crossing after being reminded

Whether to linger in the middle of the road	The one did not linger in the middle of the road	The student stays in the middle of the road, but when reminded, quickly follow instructions and moves on	The student stays in the middle of the road, but after a long reminder, reluctantly listens to the command and continues on	The student stays in the middle of the road, and after reminding still do not listen to instructions, refused to move on, and continue to linger

When crossing the road, whether to observe the left and right road conditions	Independently observe the left and right road conditions	At the beginning, the left, right, front, and back road conditions were not observed independently, but after one reminder, the left, right, front, and back road conditions were observed	At the beginning, the left, right, front, and back road conditions were not observed independently. After several reminders, the left, right, front, and back road conditions were observed	After several reminders, still do not observe the left and right road conditions

The number of times one misses a green traffic light before starting to cross the road	Not to miss the green light	Miss the green light once	Miss the green light twice	Miss the green light three times or more

Whether to run a red light		The one that did not run the red light		To run the red light

The way to cross the street		Normal frequency step speed		Walking at an unusual frequency, such as walking very slowly and running very fast for no reason

The total number of accidents		No accident		An accident

**Table 9:** What to do if lost: student learning evaluation record sheet.

Evaluation of project	Score		
	2 points	1 point	0 point
The emotional state of being lost	A little flustered at first, but soon calmed down	A little flustered and unable to calm down quickly	Extremely flustered, completely overwhelmed, and unable to calm down

The reaction to being lost	Students actively seek help from reliable people around them	After being prompted, students can ask for help from reliable people around them	After prompting, the students could not calm down and ask for help from the reliable people around them

Call for help	Students are not timid and can take the initiative to explain	After the prompts, the students can explain their own situation and issue a request for help	After being prompted, the student was still unable to explain his situation and issued a request for help

Describe personal information	Students accurately state their home or school address, and parents or teachers contact information	Students are unable to accurately state the address of their home or school, and the contact information of their parents or teachers (or are unclear)	Students have no memory of their home or school addresses, or parents or teachers' contact information

**Table 10:** Shopping: student learning evaluation record form.

Evaluation of project	Score		
	2 points	1 point	0 point
Shopping list	Students make a shopping list (or remember exactly what they need to buy)	Students did not make a shopping list, but they could remember almost all the items they needed to buy	Students did not make a shopping list and did not remember what they needed to buy

Enter the supermarket	The student should find the entrance quickly and accurately (within 10′) and queue up to enter, being polite and not disturbing others	The student spent too much time looking for the entrance (within 30′), showing some nervous performance	Unable to find the entrance (over 60′), the student is still at a loss and needs help

Choose goods	The student can choose what he needs according to the classification of supermarket goods	The student could not accurately find the location of the goods according to the classification, but he could select the goods he needed after being prompted to classify the goods in the supermarket	The student could not accurately find the location of the goods according to the classification; after being prompted, he still could not select the goods he needed according to the classification of the goods in the supermarket

Ask the shopping guide	When the product is not available, the student has the consciousness to seek help from the shopping guide	When the product is not found, the student has the consciousness to ask the shopping guide for help after being prompted	When the product cannot be found, the student goes through the prompts and does not ask the shopping guide for help

Waiting in line to pay	The student has the consciousness of waiting in line to pay	After being prompted, the student queued for payment	After being prompted, the student still did not queue up to pay

Put things in bags and return	After the payment is finished, the student will take the initiative to tidy up the items and return them to the bag	After being prompted, the student put the bought items into a bag and returned them	After being prompted, the student still did not tidy up the items in the bag

**Table 11:** Bus ride: student learning evaluation record form.

	Evaluation of project	Score		
		2 points	1 point	0 point
The first practice	Waiting in line for the bus	Take the initiative to perform tasks without prompting	Perform the task only when prompted	After being prompted, the task still cannot be executed
	Pay the ticket by card			
	Get in and find a seat			
	Ask			
	Wait until the stop prompts to get off			

The second practice	Waiting in line for the bus			
	Pay the ticket by card			
	Get in and find a seat			
	Ask			

The third practice	Wait until the stop prompts to get off			
	Waiting in line for the bus			
	Pay the ticket by card			
	Get in and find a seat			
	Ask			
	Wait until the stop prompts to get off			

**Table 12:** Interview: student learning evaluation record.

Evaluation of project	Score		
	2 points	1 point	0 point
Comfort in conversation	This person can communicate easily with the interviewer, has certain interview skills, and behaves well	Moderate comfort, with some signs of tension	Very anxious and physical symptoms

Degree of effort	Keywords: hard work, dedication, volunteer to do more, and put work first	Keywords: the person states that he will work hard but cannot give examples of what constitutes hard work and says things that are unreliable and untrustworthy; the words are inconsistent	Keywords: likely to be late for work, refusing to accept responsibility, being lazy, and unreliable

Attitude towards working with others	This person is flexible, can get along well with colleagues, helpful, willing to accept training, abide by rules, and follow arrangements	This person was generally able to get along well with colleagues, but showed some difficulties	The person criticized the boss/colleagues, had conflicts with others, and complained about some

Degree of honesty	The answer is reliable and trustworthy	He was mostly honest, but some of his answers were inconsistent	His answers are unreliable, dishonest, and untrustworthy

Degree of specialization	This person is polite (thank you and please), respectful, and treats the interviewer such as a supervisor	Some of the answers were professional but lacked polite language	The person is overly casual, overshares, and talks about issues not relevant to the interview (parties, meals, etc.)

Degree of harmony	This person is actively engaged in formal conversation, nodding when asked, smiling a lot, making eye contact, and being enthusiastic	This person shows a friendly attitude, but the conversation is not focused on work	The person pauses awkwardly, barely makes eye contact, gives short answers, and has a negative attitude

## Data Availability

The dataset can be obtained from the corresponding author upon request.
